The article "Research on the Correlation of Peripheral Blood Inflammatory Markers with PCT, CRP, and PCIS in Infants with Community-Acquired Pneumonia" was retracted in 2023. Reasons: signs of a paper mill; suspected computer-generated content; unreliable results or conclusions; concerns about the data.

# Research on the Correlation of Peripheral Blood Inflammatory Markers with PCT, CRP, and PCIS in Infants with Community-Acquired Pneumonia

**DOI:** 10.1155/2022/9024969

**Published:** 2022-10-17

**Authors:** Linwei Li, Hongyun Miao, Xue Chen, Shengjie Yang, Xiaoyong Yan

**Affiliations:** ^1^Department of Pediatrics, Jiangjin Hospital Affiliated to Chongqing University, No. 725, Jiangzhou Avenue, Dingshan Street, Jiangjin District, Chongqing, China; ^2^Department of Endocrinology, Jiangjin Hospital Affiliated to Chongqing University, No. 725, Jiangzhou Avenue, Dingshan Street, Jiangjin District, Chongqing, China

## Abstract

**Aims:**

This study aimsto investigate the relationship between peripheral blood neutrophil/lymphocyte ratio (NLR), platelet/lymphocyte ratio (PLR), systemic immune-inflammatory index (SII), and procalcitonin (PCT), C-reactive protein (CRP), and pediatric critical illness score (PCIS) in infants with community-acquired pneumonia (CAP).

**Methods:**

100 infants with bacterial CAP admitted to our hospital between January 2021 and December 2021 were selected as the infected group, and another 100 healthy infants who underwent health check-ups at the same time were selected as the control group, and the NLR, PLR, and SII of peripheral blood of infants in both groups and the serum PCT, CRP, and PCIS scores of infants in the infected group were tested. The correlation between NLR, PLR, SII, and PCT, CRP, and PCIS was analyzed by Spearman's analysis.

**Results:**

The peripheral blood levels of NLR, PLR, and SII were higher in the infected group than in the control infants (*P* < 0.05). The ROC results showed that the AUCs of peripheral blood NLR, PLR, and SII for the diagnosis of infants with CAP were 0.934, 0.737, and 0.882, respectively. The ROC results showed that the AUCs of peripheral blood NLR, PLR, and SII for assessing the extent of disease in infants with CAP were 0.815, 0.710, and 0.813, respectively, with best cut-off values of 2.05, 98.57, and 823.41; the joint predicted AUC was 0.862.

**Conclusions:**

NLR, PLR, and SII were significantly elevated in the peripheral blood of infants with CAP, positively correlated with PCT and CRP, and negatively correlated with PSIC scores, and NLR and SII also have some guiding value in early diagnosis and assessment of the extent of the disease in infants and toddlers with CAP.

## 1. Introduction

Community-acquired pneumonia (CAP) remains the most common respiratory disease in children and the leading cause of death in children under five years of age. Due to their anatomical and immunological characteristics, infants are prone to respiratory infections, and their infections spread easily, and their upper respiratory tract infections are also prone to develop into pneumonia, even severe pneumonia [1, 2]. Many factors can cause pneumonia in infants, such as pathogenic infections, poor lung development, poor environment, and care, etc. Among them, pathogenic infections (bacteria, viruses, and so on.) are the most common and can affect the growth and development of infants in severe cases [3].

Clinical studies have shown that the key to the treatment of CAP in infants lies in the early identification of the pathogen and the targeted adoption of reasonable anti-infection treatment, which can effectively improve clinical symptoms and prognosis and has important clinical significance [4]. In recent years, with the development of serological diagnostic markers, serum indicators such as procalcitonin (PCT) and C-reactive protein (CRP) have become more clinically accepted indicators to assess the status of infection, and their elevation can reflect the severity of the disease; the PCIS score is also the most objective, widely used, and effective score in China, which can effectively reflect the criticality of the child's condition and has a good predictive effect on the risk of death [5]. However, the above indexes and scores are difficult to apply in primary hospitals due to the difficulties of venous blood collection from small infants, long laboratory time, and poor generalizability. In this study, peripheral blood inflammatory markers: neutrophil/lymphocyte ratio (NLR), platelet/lymphocyte ratio (PLR), and systemic immune inflammatory index (SII, platelets × neutrophils/lymphocytes) were used to explore their correlation with blood CRP, PCT, and pediatric critical illness score (PCIS). To explore a quick, easy, and cost-effective way to assess the condition of pneumonia in infants, and to provide data and results of the research, we report the following.

The purpose of this paper is to explore the relationship between the peripheral blood neutrophil/lymphocyte ratio (NLR), platelet/lymphocyte ratio (PLR), systemic immune inflammatory index (SII), procalcitonin (PCT), C-reactive protein (CRP) and children's critical case score (PCIS) in children with community-acquired pneumonia (CAP), and to provide reference results for solutions.

## 2. Information and Methods

### 2.1. General Information

A total of 100 infants with CAP who were admitted to our hospital between January 2021 and December 2021 were selected as the infected group, and another 100 healthy infants who were examined at the same time in our child health department were selected as the control group.

#### 2.1.1. Inclusion Criteria

Infants in the study group were required to meet both (1) the diagnostic criteria of the “Diagnosis of CAP in children (2019 edition)” in all cases [6]; (2) age 29 d to 1 week of age, all full-term singleton fetuses; and (3) positive sputum bacterial culture results; infants in the control group were required to meet both (1) the health check-up infants in our pediatric clinic; and (2) age 29 d to 1 week of age, all full-term singleton fetuses.

#### 2.1.2. Exclusion Criteria

For both groups of infants, exclusion was based on any of the following: history of resuscitation by asphyxia at birth, the combination of congenital heart disease; renal disease; trauma; diabetes; hypertension; Kawasaki disease or connective tissue disease; immunodeficiency disorders; identification of extrapulmonary bacterial infections; and airway malformations. The study was approved by the hospital ethics committee; informed consent was signed by the parents of both groups of infants before enrollment. There were 55 males and 45 females in the infected group, with a mean age of (7.82 ± 2.65 months); 47 males and 53 females in the control group, with a mean age of (8.27 ± 2.30) months. The differences in basic information such as gender and age of infants in the two groups were not statistically significant (*P* > 0.05) and were comparable.

### 2.2. Methods

#### 2.2.1. Routine Blood Test

After the infants in both groups were enrolled, 5 mL of fasting venous blood was collected in the early morning, and a fully automated blood cell analyzer was applied to perform routine blood tests (neutrophil count, lymphocyte count, monocyte count, platelet count) and calculate NLR, PLR, and SII.

#### 2.2.2. Detection of Serum CRP and PCT Levels

The infants in the infected group had 4 mL of venous blood collected, and the supernatant was collected after centrifugation at 3000 r/min for 10 min at room temperature for 30 min and stored at −20°C. The serum samples were sent to Goldfield Medical Testing Center for CRP and PCT level testing.

#### 2.2.3. Severity Scores

The severity of the infant's disease was assessed by the PCIS score based on the child's vital signs, blood analysis, blood gas analysis, electrolytes, and renal function test results at the time of admission, combined with the child's digestive system symptoms and signs, in which a score of >80 indicates noncritical, 71–80 indicates critical, and ≤70 indicates very critically [7].

### 2.3. Statistical Analysis

Spearman correlation analysis is applicable to judge the correlation between two continuous variables with non-normal distribution (or with abnormal values that cannot be eliminated). When using Spearman correlation analysis, two conditions need to be met: variables are continuous variables with non-normal distribution (or with abnormal values that cannot be eliminated); and there is a monotonic relationship between variables. The IBM SPSS Statistics 22.0 statistical software was used for statistical analysis of the data, and measures that conformed to a normal distribution with homogeneous variance were expressed as mean ± standard deviation ($\bar{x}\pm s$), and independent samples *t*-test was used for comparison between groups, while measures of non-normally distributed data were expressed as [*M* (*Q*_*R*_)] and Mann–Whitney *U* test was used for comparison between groups. Count data were expressed as cases or percentages, using the chi-square test; Spearman correlation analysis was used to analyze the correlation between NLR, PLR, and SII and PCT, CRP, and PCIS indicators; The efficacy of NLR, PLR, and SII in the diagnosis of CAP and assessment of the extent of the condition in infants was assessed using the receiver operating characteristic curve (ROC), with *P* < 0.05 indicating a statistically significant difference.

## 3. Results

### 3.1. Comparison of NLR, PLR, and SII Levels in Peripheral Blood of Infants in Two Groups

The peripheral blood levels of NLR, PLR, and SII were higher in the infected children than in the control infants (*P* < 0.05). See Table 1.

### 3.2. Correlation Analysis of Peripheral Blood NLR, PLR, and SII Levels with PCT, CRP, and PCIS Scores in Infants of the Infected Group

The results showed that PCT, CRP, and PCIS were non-normally distributed in the infected group of children, with median and interquartile distances of 0.82 (1.06), 16.90 (20.8), and 100.00 (8.00), respectively. Spearman analysis showed that NLR, PLR, and SII were positively correlated with PCT and CRP (all *P* < 0.05), and PCIS scores were negatively correlated (all *P* < 0.05). See Table 2.

### 3.3. ROC Analysis of Infants with CAP Diagnosed by Peripheral Blood NLR, PLR, and SII

The ROC results showed that the AUCs of peripheral blood NLR, PLR, and SII for the diagnosis of infants with CAP were 0.934, 0.737, and 0.882, respectively. The best cut-off values based on the Jorden index were 0.54, 84.96, and 188.35, respectively. The sensitivity and specificity based on the best cut-off values were 91.00%, 84.00%, and 68.00%, and 74.00%, 86.00%, and 79.00%. See Figure 1, Table 3.

### 3.4. Comparison of Peripheral Blood Levels of NLR, PLR, and SII in Infants with Different Severity

According to the PCIS score, 12 children with scores below 80 were in the severe group and the rest were in the mild group. The blood NLR, PLR, and SII levels of children in the mild group were lower than those in the severe group (*P* < 0.05). See Table 4.

The ROC results showed that the AUCs of peripheral blood NLR, PLR, and SII for predicting the extent of disease in infants with CAP were 0.815, 0.710, and 0.813, respectively. The sensitivity and specificity based on the best cut-off values were 91.67%, 62.50%, and 91.67%, 51.95%, 91.67%, and 64.77%. Based on the coefficients obtained from logistic regression to establish the joint detection index, the AUC of the joint detection was 0.862, and the sensitivity and specificity were 100% and 69.32%, respectively, which were higher than the prediction alone. See Table 5, Figure 2.

## 4. Discussion

Pneumonia is the leading cause of death in children under 5 years old in China, the vast majority of whom are CAP, and bacterial infection is the leading cause of CAP [7]. Once an infection occurs in infants and young children under 2 years old, it can easily develop into bronchitis or bronchopneumonia, or even severe pneumonia, posing a serious threat to the health of infants and toddlers [8]. The main clinical difficulties are the differentiation from noninfectious diseases and the clarification of the pathogenic diagnosis of infants who have failed empirical treatment. Although the sputum smear technique is faster, it requires high sputum samples, and even after the initial identification of pathogenic species, a further sputum culture is still needed to clarify the pathogenic bacteria, while blood culture is only applicable to bacterial lung infections with bacteremia, and its clinical use is more limited, so it is clinically important to find some laboratory indicators for early diagnosis, disease assessment, and prognosis of bacterial pneumonia in infants.

The indicators currently included in the guidelines for CAP evaluation are leukocyte-to-neutrophil ratio, CRP, and PCT, but the sensitivity and specificity of these indicators for clinical application are still unsatisfactory [9]. Cellular immune dysfunction and disorders are the most studied pathogenesis of CAP in addition to the direct pathogen invasion theory [10]. Leukocytes and their subtypes (monocytes, lymphocytes, and macrophages), as important immune cells involved in immune regulation, can cause changes in the level of relevant immune cells in the body when bacteria enter the body, and NLR, PLR, SII, and so on are important indicators reflecting the inflammatory response in the body obtained based on the level of immune cells [11–13]. In this study, 100 infants under 1 year of age diagnosed with bacterial CAP were selected as the infected group, and 100 healthy infants were selected as the control group during the same period. The levels of NLR, PLR, and SII in the peripheral blood of the two groups were compared, and it was found that the levels of NLR, PLR, and SII in the peripheral blood of the infected infants were significantly higher than those of the control infants. As an important indicator of the inflammatory response and immune homeostasis, the level of NLR in the peripheral blood of infants with bacterial CAP was significantly higher, which was consistent with the findings of Jiang et al. [14]; altered coagulation also plays an important role in the inflammatory response, but the body releases a variety of cytokines after infection, which activate the coagulation system and inhibits the fibrinolytic system. The PLR, as a ratio of platelet to lymphocyte levels, has higher stability compared to the two alone, and thus, PLR levels were significantly higher, in line with the findings of Lu and Zhu [15]; SII is an index that comprehensively reflects the inflammatory and immune homeostasis status of the body, calculated by platelet count, neutrophil, and lymphocyte levels, and the activation of immune function and inflammatory response caused by pathogen invasion can cause a significant increase in SII levels, in agreement with the findings of Acar et al. [16].

To further investigate the clinical application value of NLR, PLR, and SII, this study compared the correlation of NLR, PLR, and SII with the traditional inflammatory indexes CRP and PCT and the PCIS score, which reflects the degree of pediatric disease, using the Spearman's correlation analysis. The results showed that NLR, PLR, and SII were positively correlated with CRP and PCT, and the correlation coefficients of NLR and SII were close to 0.8, suggesting that these three may have a high diagnostic value. The results of ROC analysis showed that the AUCs of NLR, PLR, and SII in the diagnosis of infants with bacterial CAP were 0.934, 0.737, and 0.882, respectively, indicating that both NLR and SII have high diagnostic value and are worthy of clinical reference. The PCIS score is an evaluation system used to reflect the systemic organ status of infants with pneumonia that is unique to our country [17]. The results of the present study showed that NLR, PLR, and SII were negatively correlated with PCIS scores, indicating that high levels of NLR, PLR, and SII may be related to the severity of disease and prognosis of an infant with CAP. By comparing the peripheral blood NLR, PLR, and SII levels of children in the severe and mild disease groups, we found that the NLR, PLR, and SII levels of children in the severe disease group were significantly higher than those in the mild disease group. The AUCs of NLR, PLR, and SII in the assessment of the severity of bacterial CAP children were found to be 0.815, 0.710, and 0.813, respectively, by ROC analysis. It indicated that NLR, PLR, and SII can differentiate the severity of CAP children, which is conducive to the timely adoption of appropriate therapeutic measures to improve the treatment effect, and the joint prediction of the three indicators is better.

## 5. Conclusions

NLR, PLR, and SII are significantly elevated in the peripheral blood of infants with CAP. As simple and easily accessible indicators for clinical work, these indicators help in the initial diagnosis and assessment of the condition of children with CAP, provide early warning information, guide active and effective clinical interventions, and play a positive role in avoiding the development of severe disease and reducing the death rate of infants and children. However, this study is a single-center, small-sample study limited to bacterial CAP, and its value in other pathogenic infection types of pneumonia requires a multicenter, larger sample randomized controlled study to further confirm the clinical credit value of the indicators in this study.

## Figures and Tables

**Figure 1:** ROC curves of peripheral blood NLR, PLR, and SII for the diagnosis of infants with CAP.

**Figure 2:** ROC curves of peripheral blood NLR, PLR, SII, and joint prediction of the extent of disease in infants with CAP.

**Table 1:** Comparison of peripheral blood NLR, PLR, and SII levels between two groups of infants [*M* (*Q*_*R*_)].

Groups	Number of cases	NLR	PLR	SII
Infection group	100	1.96 (1.71)	98.91 (33.60)	739.04 (898.79)
Control group	100	0.32 (0.21)	69.39 (34.05)	119.34 (99.43)
*Z*		10.609	5.796	9.341
*P*		<0.001	<0.001	<0.001

**Table 2:** Correlation analysis of peripheral blood NLR, PLR, and SII levels with PCT, CRP, and PCIS scores.

	NLR		PLR		SII	
	*r*	*P*	*r*	*P*	*r*	*P*
PCT (ng/mL)	0.798	<0.001	0.488	<0.001	0.788	<0.001
CRP (mg/L)	0.760	<0.001	0.493	<0.001	0.763	<0.001
PCIS (scores)	−0.568	<0.001	−0.348	<0.001	−0.595	<0.001

**Table 3:** Efficacy of peripheral blood NLR, PLR, and SII in the diagnosis of infants with CAP.

Index	AUC	Best cut-off values	95% CI confidence interval	Sensitivity (%)	Specificity (%)
NLR	0.934	0.54	0.890∼0.964	91.00	84.00
PLR	0.737	84.96	0.670∼0.797	68.00	74.00
SII	0.882	188.35	0.829∼0.923	86.00	79.00

**Table 4:** Comparison of peripheral blood levels of NLR, PLR, and SII in infants with different severity [*M* (*Q*_*R*_)].

Groups	Number of cases	NLR	PLR	SII
Severe group	12	2.84 (1.60)	126.76 (42.93)	1249.78 (497.10)
Mild group	88	1.72 (1.57)	95.11 (30.50)	624.43 (824.80)
*Z*		3.538	2.355	3.500
*P*		<0.001	<0.05	<0.001

2.5 ROC analysis of peripheral blood NLR, PLR, and SII to assess the extent of disease in infants with CAP.

**Table 5:** Efficacy of peripheral blood NLR, PLR, and SII in diagnosing the extent of disease in infants with CAP.

Index	AUC	Best cut-off values	95% CI confidence interval	Sensitivity (%)	Specificity (%)
NLR	0.815	2.05	0.708∼0.923	91.67	62.50
PLR	0.710	98.57	0.583∼0.837	91.67	51.95
SII	0.813	823.41	0.715∼0.910	91.67	64.77
Joint forecast	0.862		0.782∼0.942	100	69.32

## Data Availability

The experimental data used to support the findings of this study are available from the corresponding author upon request.
